The article "Analysis of the Effectiveness of the Nurse-Led “Outpatient-Ward-Home” Management Model in Chronic Kidney Patients" was retracted in 2023. Reasons: signs of a paper mill; suspected computer-generated content; unreliable results or conclusions; concerns about the data.

# Analysis of the Effectiveness of the Nurse-Led “Outpatient-Ward-Home” Management Model in Chronic Kidney Patients

**DOI:** 10.1155/2022/4229436

**Published:** 2022-09-30

**Authors:** Qi Hu, Xue Yang, Wei Wang, Man Meng

**Affiliations:** ^1^Nephrology Internal Medicine Ward, The First Affiliated Hospital of Jinzhou Medical University, Jinzhou, Liaoning 121000, China; ^2^General Surgery (Large Intestine) Ward 1, The First Affiliated Hospital of Jinzhou Medical University, Jinzhou, Liaoning 121000, China; ^3^Endocrinlology and Metabolic Diseases Ward, The First Affiliated Hospital of Jinzhou Medical University, Jinzhou, Liaoning 121000, China

## Abstract

**Objective:**

To investigate the application and effect of the nurse-led “outpatient-ward-home” management model in the care of patients with chronic kidney disease (CKD).

**Methods:**

120 patients with CKD admitted to our hospital between April 2020 and April 2021 were selected as trial subjects. All patients were divided into experimental and control groups according to the random number table method, with 60 cases in each group. The patients in the experimental group implemented the nurse-led “outpatient-ward-home” management model; the patients in the control group were given routine care and telephone follow-up. The self-rating anxiety scale (SAS), self-rating depression scale (SDS), Pittsburgh Sleep Quality Index (PSQI) score, self-management scores, nutritional status, renal function indicators, and chronic renal failure quality of life scale (QLICD-CRF2.0) were compared between the two groups before and 6 months after the intervention.

**Results:**

Before the intervention, there were no statistically significant differences between the control and experimental groups in SAS, SDS, PSQI scores, self-management scores, QLICD-CRF2.0 scores, body mass index (BMI), prealbumin (PAb), albumin (ALB), serum creatinine (Scr), blood urea nitrogen (BUN), and glomerular filtration rate (GFR) levels (*P* > 0.05). After 6 months of intervention, SAS, SDS, PSQI scores, Scr, BUN, and GFR levels were lower in the experimental group than in the control group; self-management scores, QLICD-CRF2.0 scores, BMI, PAb, and ALB levels were higher in the experimental group than in the control group (*P* < 0.05).

**Conclusion:**

The nurse-led “outpatient-ward-family” intervention model can improve the negative emotions and sleep disorders of CKD patients, enhance patients' self-management ability, and to a certain extent, slow down the disease process and improve the quality of life.

## 1. Preface

Chronic kidney disease (CKD) is a progressive clinical syndrome of chronic renal structural and functional disorders caused by various causes, with an insidious early onset, often accompanied by chronic diseases such as diabetes and hypertension, and an irreversible course, eventually developing into end-stage renal disease [1, 2]. A related study [3] showed that the effective treatment of CKD in China is only 7.5% due to the lack of adequate knowledge of the disease, low self-management ability, and the constraints of the current health insurance reimbursement system. The progression of CKD patients is closely related to their lifestyles, and improving patients' self-management ability is the key to slow down the progression of their disease. Related studies [4, 5] showed that the self-management ability of CKD patients is at an intermediate level, and there is still much room for improvement. An effective disease treatment management model is a prerequisite for slowing disease progression, improving patient adherence to treatment, maintaining disease stability, improving patient quality of life, reducing patient health care costs, and promoting the doctor-patient relationship [6]. At present, the management model of CKD patients in China lacks consistency, comprehensiveness, and systematization, which leads to poor patient compliance with treatment and further results in accelerated loss of renal function, so consistent and comprehensive management of patients on the basis of conventional treatment is also needed. The single ward education model is simple and has low acceptance by patients, so it is necessary to carry out the whole process of nursing management for CKD patients by integrating the application of previous nursing models.

The article "Analysis of the Effectiveness of the Nurse-Led “Outpatient-Ward-Home” Management Model in Chronic Kidney Patients" was retracted in 2023. Reasons: signs of a paper mill; suspected computer-generated content; unreliable results or conclusions; concerns about the data.

It has been shown that a CKD management team combined with integrated community management can effectively improve renal function, delay disease progression and improve the quality of life in patients with CKD [7, 8]. Several studies [9–11] have shown that integrated outpatient-ward-family management improves fear, depression, anxiety, and sleep disturbances in patients with mild cognitive impairment, hypertension, and stroke. In this study, on the basis of the previous routine continuing care, according to the clinical characteristics of CKD patients, the whole process nursing model based on the ward-outpatient-family was implemented. However, considering the lack of professional knowledge and support experience of patients and their families, they often need professional guidance from healthcare professionals. There are few reports in the literature on how nurses, as the main body of nursing care in China, can play a better role in the nursing management of CKD through nurse-led outpatient-ward-family. In this paper, we constructed a nurse-led outpatient-ward-family intervention model to manage CKD patients in all aspects of the ward, outpatient clinic, and family, and observed the effects of the model on the self-management ability and nutritional status of CKD patients, aiming to provide a reference basis for improving the survival quality of CKD patients.

The article "Analysis of the Effectiveness of the Nurse-Led “Outpatient-Ward-Home” Management Model in Chronic Kidney Patients" was retracted in 2023. Reasons: signs of a paper mill; suspected computer-generated content; unreliable results or conclusions; concerns about the data.

## 2. Data and Methods

### 2.1. General Data

120 patients with CKD admitted to our hospital between April 2020 and April 2021 were selected as the test subjects. According to the random number table method, all patients were divided into an experimental group and a control group, with 60 patients in each group. The patients in the experimental group implemented the nurse-led “ward-outpatient-family” management model; the patients in the control group were given routine care and telephone follow-up. Inclusion criteria were as follows: (i) all of them fulfilled the relevant CKD diagnostic criteria of the CKD clinical practice guidelines (K/DOKI) [12]. (ii) patients without serious organ disease; (iii) patients who were conscious and able to cooperate with the study; (iv) clinical stage I to III; (v) aged ≥ 18 years. Exclusion criteria were as follows: (i) those with combined mental illness or cognitive dysfunction; (ii) those with hearing or visual impairment affecting normal communication; (iii) the presence of serious comorbidities.

### 2.2. Intervention Methods

#### 2.2.1. Control Group (Conventional Nursing Intervention)

*(1) On Admission*. Patients were promptly given an admission health assessment upon admission; the nurse-in-charge conducted bedside education, including an introduction to the nurse-in-charge, supervising physician and ward environment; and answered patients' questions.

*(2) During Hospitalization*. (i) Basic nursing care: included ward environment organization, medication, and patient safety. (ii) Specialist nursing care: edema care, renal puncture care, notification of 24 h urine specimen retention method, etc. (iii) Group lectures: included diet, medication, activity, and other kidney disease-related knowledge, once/week. (iv) Playing video: half-hour video related to kidney diet, medication, and other precautions is played in the nursing check-in car every morning. (v) Regular rounds: the responsible nurse regularly rounded the patients according to the nursing classification and solved patients' problems at any time; (vi) Psychological care: nurses took the initiative to care for and pay attention to the emotional changes of patients, and provided psychological guidance when necessary.

*(3) At the Time of Discharge*. (i) Informed patients of the precautions to be taken after discharge, including taking medication according to medical advice, reasonable diet, regular monitoring of blood glucose, and blood pressure; (ii) issued the hospital's homemade CKD health management manual and salt spoon, reconfirmed with patients the time of review, and instructed patients to come to the hospital for review as prescribed by the doctor; (iii) made routine telephone follow-up visits; (iv) informed patients of the telephone numbers of nurses' stations and doctors' offices, and encouraged patients to consult if they had any questions.

The article "Analysis of the Effectiveness of the Nurse-Led “Outpatient-Ward-Home” Management Model in Chronic Kidney Patients" was retracted in 2023. Reasons: signs of a paper mill; suspected computer-generated content; unreliable results or conclusions; concerns about the data.

#### 2.2.2. Experimental Group

*(1) Formation of a Nurse-Led Family Support Intervention Group*. The head nurse served as the group leader, and the members included the department head, responsible doctors, nurses, rehabilitation workers, and dieticians. Developed a group management system and division of responsibilities to provide a strong guarantee for the implementation of the care program.

*(2) Outpatient Management*. The CKD clinic was attended by one CKD specialist nurse daily to establish personal files and conduct a systematic assessment for patients with CKD on their first visit and to inform the department to prepare patients for admission. We provided guidance on oral medication management, self-monitoring, lifestyle, rehabilitation activities, nutritional management, and rest and sleep for repeat patients, as well as health education on risk factors and triggering factors.

*(3) Ward Management*. (i) Upon admission, physicians promptly assessed the condition and negative emotions of CKD patients, gave timely standardized treatment and health education, and promptly relieved patients' adverse emotions. (ii) Psychological guidance: The responsible nurse analyzed the reasons for the negative emotions of patients through selective in-depth interviews with hospitalized patients and eliminated the negative emotions of patients towards the disease through encouragement, comfort, and communication. (iii) Health education: Patients were allowed to watch disease-related science videos on mobile TV for a limited period of time, nurses provided disease-related pamphlets and health education prescriptions, and for patients with end-stage CKD, nurses used specific food models to educate patients on the types and amounts of foods that were healthy for CKD disease. (iv) Nutritional intervention: Based on the patient's condition, biochemical indicators, blood pressure, dietary habits, family economic strength, etc., the deployment of a targeted and reasonable diet, as chronic kidney disease could lead to malnutrition, which in turn resulted in the decline of the patient's immunity, so it was also necessary to ensure a reasonable intake of protein.

*(4) Home Management Multiform and Multichannel Implementation of Postdischarge Extended Care and Follow-Up Guidance*. (i) Set up a CKD discharge patient care Weibo group to answer questions and solve problems for discharged patients, regularly push relevant disease rehabilitation knowledge and self-management knowledge, and provide psychological support and emotional guidance. (ii) WeChat follow-up: follow-up at day 3, 2 weeks, 4 weeks, 6 weeks, 8 weeks, and 12 weeks after discharge, with more frequent follow-ups according to patients' needs. In accordance with the follow-up plan and content formulated before discharge, patients were given priority for video follow-up by WeChat, supplemented by QQ, telephone, and SMS. Dynamically understood patients' condition recovery and self-management, asked patients about their objective data related to subjective feelings and self-monitoring, and understood patients' drug efficacy, adverse reactions, and dose adjustment plan. Patients' medication taking, self-monitoring, and rehabilitation exercise compliance were evaluated, self-management goals were checked via video and follow-up rehabilitation plans were made, appointments were made for next communication and follow-up visits, and follow-up records were made. Problems raised by patients during the follow-up visit, such as treatment, rehabilitation, and nutrition, were fed back to team members by the follow-up specialist nurse on the same day, and targeted guidance was provided by dedicated staff. (iii) Regularly carry out doctor-patient association meetings: the patients in the experimental group held a renal friend meeting once every 2 months, at which renal disease medical experts were invited to answer various problems encountered by the patients in the treatment, to provide targeted treatment and mental support to patients, and to increase the interaction between doctors and patients and nurses and patients.

The article "Analysis of the Effectiveness of the Nurse-Led “Outpatient-Ward-Home” Management Model in Chronic Kidney Patients" was retracted in 2023. Reasons: signs of a paper mill; suspected computer-generated content; unreliable results or conclusions; concerns about the data.

### 2.3. Evaluation Indexes

Socio-demographic data such as patient age, gender, marital status, medical payment method, per capita monthly household income, and body mass index (BMI) were collected by reviewing patients' medical records. Disease-related information such as primary disease, disease duration, CKD stage, comorbidities or complications, number of hospitalizations, blood pressure (BP), serum creatinine (Scr), blood urea nitrogen (BUN), prealbumin (PAb), albumin (Alb), and glomerular filtration rate (GFR). Before and after 6 months of intervention, patients' Self-Rating Anxiety Scale (SAS) [13], Self-rating depression scale (SDS) [14], Pittsburgh Sleep Quality Index (PSQI) [15], self-management behavior, and quality of life were compared. The team nurses interpreted the entries of all the above scales for the patients one by one, and for patients with low literacy levels who could not fill out the forms independently, their family members filled them out on their behalf, and all the scales were distributed and collected on the spot.

(i) The SAS was used to assess the anxiety status of patients. The SAS was scored according to the SAS Chinese norm, and the SAS score was 1∼100. The higher the score, the higher the level of anxiety. 50–59 indicated mild anxiety, 60–69 was moderate anxiety, and 69 or more was severe anxiety. (ii) SDS was used to assess patients' depression status, and the SDS score was 1∼100. The higher the score, the more severe the depression. 53–62 was mild depression, 63–72 was moderate depression, and greater than 72 was severe depression. (iii) Sleep quality: the PSQI was used to assess the sleep quality of patients, with a PSQI score of 0–21. The higher the score, the worse the sleep quality. 0∼5 was very good sleep quality, 6∼10 was good sleep quality, 11∼15 was fair sleep quality, and 16∼21 was very poor sleep quality. (iv) Self-management behavior: the self-management scale for chronic kidney patients developed by Yu Ping et al. was used, with a Cronbach's alpha coefficient of 0.902. The scale had 31 items with 4 dimensions, namely: dietary management, therapeutic management, physical activity management, and psychosocial management. Each item was scored on a scale of 1 to 4, with a total score of 124, with higher scores indicating better self-management behavior. (v) Quality of life: the chronic kidney disease quality of life measurement scale (QLICD-CRF2.0) was used, which consists of 4 dimensions: psychological functioning (0–55 points), physical functioning (0–35 points), social relationships (0–20 points), and treatment status (0–20 points), with a total of 27 entries. The evaluation criterion was that higher scores indicated better quality of survival. (vi) Laboratory index tests: SCr, BUN and CysC, PAb, and ALB were performed at the time of discharge and 6 months after discharge, along with BMI measurement.

### 2.4. Data Analysis

The data were numbered, entered into an Excel sheet by the investigator and another person unrelated to this study, and double-checked, and SPSS 21.0 was used to analyze the data. Mean ± SD, median, and interquartile spacing were used for measurement data, and frequency and percentage were used for count data; for comparison of baseline data between the two groups, the chi-square test was used for count data, and *t*-test and nonparametric test for two independent samples were used for measurement data. *P* < 0.05 was considered a statistically significant difference.

The article "Analysis of the Effectiveness of the Nurse-Led “Outpatient-Ward-Home” Management Model in Chronic Kidney Patients" was retracted in 2023. Reasons: signs of a paper mill; suspected computer-generated content; unreliable results or conclusions; concerns about the data.

## 3. Results

### 3.1. Comparison of General Information of Patients in the Two Groups

By reviewing the patients' medical history data including patients' age, gender, marital status, and per capita monthly income, and the disease-related data including primary disease, disease duration, CKD stage, and the number of comorbidities or complications, and conducting statistical analysis of the collected data in groups, the results showed that there was no statistically significant difference between the two groups in the above general data (*P* > 0.05), as shown in Table 1.

### 3.2. Comparison of Psychological Status and Sleep Quality between the Two Groups of Patients before and after 6 Months of Intervention

Before the nursing intervention, the comparison of SAS, SDS, and PSQI scores between the control group and the experimental group was not significant (*P* > 0.05). After 6 months of intervention, the SAS, SDS, and PSQI scores of the experimental group were significantly lower than those of the control group, and the difference was statistically significant (*P* < 0.05). See Figure 1 for details.

### 3.3. Comparison of Self-Management Scores between the Two Groups before and after 6 Months of Intervention

The differences between the control and experimental groups were not significant (*P* > 0.05) when comparing the dietary management, therapeutic management, physical activity management, and psychosocial management scores before the nursing intervention. After 6 months of intervention, the dietary management, therapeutic management, physical activity management, and psychosocial management scores of the experimental group were significantly higher than those of the control group, and the difference was statistically significant (*P* < 0.05). See Figure 2 for details.

### 3.4. Comparison of the Nutritional Status of Patients in the Two Groups before and after 6 months of Intervention

Before the nursing intervention, the PAb, ALB, and BMI levels of the control group were not significantly different from those of the experimental group (*P* > 0.05). After 6 months of intervention, the PAb, ALB, and BMI levels of the experimental group were significantly higher than those of the control group, and the differences were statistically significant (*P* < 0.05). See Figure 3 for details.

### 3.5. Comparison of Renal Function Indexes between the Two Groups of Patients before and after 6 Months of Intervention

Before the nursing intervention, the levels of Scr, BUN, and GFR in the control group and the experimental group were not significantly different from each other (*P* > 0.05). After 6 months of intervention, the levels of Scr, BUN, and GFR in the experimental group were significantly lower than those in the control group, and the difference was statistically significant (*P* < 0.05). See Figure 4 for details.

The article "Analysis of the Effectiveness of the Nurse-Led “Outpatient-Ward-Home” Management Model in Chronic Kidney Patients" was retracted in 2023. Reasons: signs of a paper mill; suspected computer-generated content; unreliable results or conclusions; concerns about the data.

### 3.6. Comparison of the Quality of Life of the Two Groups before and after 6 Months of Intervention

The differences between the control group and the experimental group were not significant (*P* > 0.05) when comparing the scores of psychological function, physical function, social relationship, and treatment status before the nursing intervention. After 6 months of intervention, the scores of psychological function, physical function, physiological function, and treatment condition in the experimental group were significantly higher than those in the control group, and the difference was statistically significant (*P* < 0.05). See Figure 5 for details.

## 4. Discussion

As a common clinical chronic disease, CKD can involve all systems of the body, and the disease is prolonged, which predisposes patients to a series of adverse emotions such as anxiety and depression [16, 17]. Laffin and Bakris [18] found that the use of integrated individualized ward-clinic-home health care management met patients' needs for all 3 aspects of treatment, care, and family and effectively reduced negative patient emotions. This paper examines the effects of integrated outpatient-ward-home healthcare management on negative emotions, sleep disorders, self-management ability, nutritional status, renal function, and quality of life in patients with CKD, with the aim of exploring ways to improve treatment compliance and quality of life in patients with CKD.

### 4.1. The Nurse-Led “Outpatient-Ward-Home” Intervention Model Improves Negative Emotions and Sleep Quality in CKD Patients

The results of this study showed that after 6 months of intervention, the experimental group showed greater reductions in SAS, SDS, and PSQI scores than the control group (*P* < 0.05). Suggesting that the integrated ward-clinic-family management model improves negative emotions and sleep quality in patients with CKD, in line. Llewellyn's [19] study results are more consistent. Because of the long-term chronic spiral progression of CKD patients, they require not only long-term repeated hospitalization but also long-term outpatient follow-up and home management. In the integrated management model of outpatient-ward-home, the responsible nurses analyze the causes of negative emotions through interviews and assessments of patients' conditions, so that patients can get comprehensive guidance such as systematic drug treatment, exercise, nutrition intake, and psychological counseling in the whole process. And a multidimensional and perfect social support network was constructed, and patients established confidence in controlling the disease, which led to the timely and effective relief of negative emotions while reducing patients' worries about the prognosis of the disease and allowing them to relax physically and mentally, which could improve their sleep disorders and improve their sleep quality [20, 21].

The article "Analysis of the Effectiveness of the Nurse-Led “Outpatient-Ward-Home” Management Model in Chronic Kidney Patients" was retracted in 2023. Reasons: signs of a paper mill; suspected computer-generated content; unreliable results or conclusions; concerns about the data.

### 4.2. The Integrated Outpatient-Ward-Home and Management Model can Improve the Self-Management Ability and Nutritional Status of CKD Patients

In this study, the BMI, PAb, and ALB of patients in the experimental group were significantly higher than those in the control group after 6 months of intervention (*P* < 0.05), indicating that the integrated outpatient-ward-home, management model can effectively improve the nutritional status of patients. This is due to the fact that healthcare education and nursing nutritional guidance intervention can promptly understand the inner conflicts of patients, develop a healthy diet plan, reasonably allocate nutrition, change patients' poor lifestyles, and promote the improvement of their nutritional status. The results showed that the self-management scores of patients in both groups improved after 6 months of intervention, and the test group was higher than the control group (*P* < 0.05), indicating that the nursing nutrition guidance intervention could effectively improve patients' self-behavior management ability, and patients could consciously change to healthier behaviors so that patients could actively cooperate with treatment. Through health education and nutritional guidance interventions, patients can also understand the knowledge and treatment methods of CKD, so that they can follow the doctor's advice; Healthy and reasonable diet control and regular exercise can improve health through behavior change [22].

### 4.3. The Integrated Outpatient-Ward-Home and Management Model can Improve the Renal Function and Quality of Life of CKD Patients

The main clinical manifestation of CKD patients is reduced renal function, and BUN, Scr, and GFR are effective indicators to detect renal function. Some studies [23, 24] have shown that lifestyle changes and dietary control of patients can improve their clinical and biochemical indicators and that this effect is independent of the effect of drug therapy. Therefore, enhancing patient self-management through active and effective interventions during the progression of CKD patients can equally influence the disease progression and outcome. In this study, there were no statistically significant differences in BUN, SCr, and GFR between the two groups before the intervention; after receiving the patients in the control group, they were given conventional care with postdischarge telephone follow-up, and the experimental group adopted the nurse-led integrated outpatient-ward-home, model. Mainly by going into the wards and families to publicize the treatment and care of the disease, making detailed follow-up plans, prioritizing the use of WeChat videos to remind patients of outpatient review, regular medication guidance to avoid the use of nephrotoxic drugs, and multidisciplinary nursing experts to develop personalized diet recipes for different patients. The problems of treatment, rehabilitation, and nutrition raised by the patients during the follow-up period were fed back to the team members by the follow-up specialist nurse on the same day, and targeted guidance was provided by the specialist to control the progress of the disease so that the patients could achieve standardized medical care and live happily [25, 26]. The results of this study showed that the differences in BUN, SCr, GFR, and quality of life between the two groups of patients after 6 months of nursing intervention were statistically significant. The nurse-led ward-outpatient-home intervention model can guide patients in a multifaceted way, help patients establish good self-management behaviors, and delay disease progression to a certain extent, which is a new nursing model with practical significance for the management of patients with chronic diseases.

The article "Analysis of the Effectiveness of the Nurse-Led “Outpatient-Ward-Home” Management Model in Chronic Kidney Patients" was retracted in 2023. Reasons: signs of a paper mill; suspected computer-generated content; unreliable results or conclusions; concerns about the data.

In conclusion, the nurse-led outpatient-ward-home, intervention model can improve the negative emotions and sleep disorders of CKD patients, enhance patients' self-management ability, and to a certain extent can delay the disease process and improve the quality of life of patients. Since the follow-up period of this study was 6 months, it did not reflect the long-term intervention effect. It is necessary to extend the follow-up period in the future, so as to comprehensively evaluate the effect of the ward-outpatient-family intervention model in patients with CKD and achieve the purpose of improving patients' health outcomes.

## Figures and Tables

**Figure 1:** Comparison of psychological status and sleep quality between the two groups of patients before and after 6 months of intervention. Note: (a) to (c) indicate the SAS score, SDS score, and PSQI score, respectively. Compared with the control group in the same period, ^*∗*^*P* < 0.05.

**Figure 2:** Comparison of self-management scores between the two groups before and after 6 months of intervention. Note: (a)∼(d) represents the score of food management, treatment management, somatic activity, and psychosocial, respectively. Compared with the control group in the same period, ^*∗*^*P* < 0.05.

The article "Analysis of the Effectiveness of the Nurse-Led “Outpatient-Ward-Home” Management Model in Chronic Kidney Patients" was retracted in 2023. Reasons: signs of a paper mill; suspected computer-generated content; unreliable results or conclusions; concerns about the data.

**Figure 3:** Comparison of the nutritional status of patients in the two groups before and after 6 months of intervention. Note: (a)∼(c) represent PAb, ALB, and BMI levels, respectively. Compared with the control group in the same period, ^*∗*^*P* < 0.05.

**Figure 4:** Comparison of renal function indexes between the two groups of patients before and after 6 months of intervention. Note: (a) to (c) represent Scr, BUN, and GFR levels, respectively. Compared with the control group in the same period, ^*∗*^*P* < 0.05.

**Figure 5:** Comparison of the quality of life of the two groups before and after 6 months of intervention. Note: (a)∼(d) represent psychological function, physical function, social relation, and treatment status score, respectively. Compared with the control group in the same period, ^*∗*^*P* < 0.05.

**Table 1:** Comparison of general information of CKD patients in two groups.

Information	Control group (*n* = 60)	Experimental group (*n* = 60)	*t*/*χ*^2^ value	*P* value
Gender (male/female)	41/19	39/21	0.150	0.699
Age (years)	46.87 ± 6.45	47.13 ± 6.22	0.225	0.823
Duration of illness (months)	22.15 ± 4.14	23.06 ± 3.97	1.229	0.222
Whether working (yes/no)	26/34	23/37	0.310	0.577
Marriage (unmarried/married)	52/8	54/6	0.324	0.570

Education level				
Primary school and below	11 (18.33)	13 (21.67)	0.546	0.909
Junior high school	28 (46.67)	25 (41.67)		
High school	13 (21.67)	15 (25.00)		
College and above	8 (13.33)	7 (11.66)		

Primary disease				
Glomerulonephritis	18 (30.00)	19 (31.67)	0.163	0.983
Hypertensive nephropathy	16 (26.67)	15 (25.00)		
Diabetic nephropathy	19 (31.67)	20 (33.33)		
Others	7 (11.67)	6 (10.00)		

Disease staging				
Stage I	28 (46.67)	30 (50.00)	0.136	0.934
Stage II	19 (3.66)	18 (30.00)		
Stage III	13 (21.67)	12 (20.00)		

Monthly income per capita (yuan)				
≤1000	18 (30.00)	20 (33.33)	0.174	0.917
1001∼3000	32 (53.33)	31 (51.67)		
≥3001	10 (16.67)	9 (15.00)		

Complications				
None/1 kind	13 (21.67)	15 (25.00)	0.220	0.896
2 kinds	27 (45.00)	25 (41.67)		
3 or more	20 (33.33)	20 (33.33)		

## Data Availability

The raw data behind the study are available upon reasonable request.
